# Genetic Analysis and Molecular Identification of Virulence in *Xanthomonas oryzae* pv. *oryzae* Isolates

**DOI:** 10.1155/2013/160157

**Published:** 2013-09-08

**Authors:** Amos Onasanya, R. O. Onasanya, Abiodun A. Ojo, B. O. Adewale

**Affiliations:** ^1^Department of Chemical Sciences, College of Sciences, Afe Babalola University, PMB 5454, Ado Ekiti, Nigeria; ^2^Federal College of Agriculture Ibadan, PMB 502, Ibadan, Nigeria

## Abstract

Bacterial leaf blight (BLB) of rice is a very destructive disease worldwide and is caused by *Xanthomonas oryzae *pv. *oryzae *(*Xoo*). The aim of the present study was to examine if the *Xoo* virulence pathotypes obtained using phenotypic pathotyping could be confirmed using molecular approach. After screening of 60 Operon primers with genomic DNA of two *Xoo* isolates (virulent pathotype, *Vr*, and mildly virulent pathotype, *MVr*), 12 Operon primers that gave reproducible and useful genetic information were selected and used to analyze 50 *Xoo* isolates from 7 West African countries. Genetic analysis revealed two major *Xoo* virulence genotypes (*Mta* and *Mtb*) with *Mta* having two subgroups (*Mta1* and *Mta2*). *Mta1* (*Vr1*) subgroup genotype has occurrence in six countries and *Mta2* (*Vr2*) in three countries while *Mtb* genotype characterized mildly virulence (*MVr*) *Xoo* isolates present in five countries. The study revealed possible linkage and correlation between phenotypic pathotyping and molecular typing of *Xoo* virulence. *Xoo* virulence genotypes were known to exist within country and there was evidence of *Xoo* pathogen migration between countries. Durable resistance rice cultivars would need to overcome both *Mta* and *Mtb Xoo* virulence genotypes in order to survive after their deployment into different rice ecologies in West Africa.

## 1. Introduction

Rice is perhaps the most widely cultivated food crop world over, but its production is constrained by diseases of fungal, bacterial, and viral origins. Bacterial leaf blight (BLB) of rice, caused by *Xanthomonas oryzae *pv. *oryzae* (*Xoo*) is a very destructive disease and its incidence has been reported from different parts of Asia, northern Australia, Africa, and USA [1–3]. The disease is known to occur in epidemic proportions in many parts of the world, incurring severe crop loss of up to 50% [1, 2, 4]. In West Africa, disease incidence ranged from 70 to 85% and yield loss ranged from 50 to 90%, indicating a wide spread of BLB disease in farmers' fields [2, 4]. Some selected *Xoo* isolates have shown high level of pathogenicity and virulence on the cultivated rice varieties [4]. Research studies have also revealed that BLB is an important rice disease in irrigated rice ecosystems in West Africa, mainly in Sahelian and Sudano-Sahelian countries [2, 5]. Crop loss assessment studies have revealed that this disease reduces grain yield to varying levels, depending on the stage of the crop, degree of cultivar susceptibility, and, to a great extent, the conduciveness of the environment in which it occurs [6]. The severity and significance of damage caused by infection have necessitated the development of strategies to control and manage the disease, so as to reduce crop loss and to avert an epidemic. Though the use of Bordeaux mixture, antibiotics, and other copper and mercurial compounds were resorted to in the early fifties, environmentally safe and stable chemical control agents rendering control at very low concentrations are yet to be developed [7]. Today, the exploitation of host resistance appears to be the only reliable method of disease management. The identification and characterization of major genes for qualitative resistance and polygenic factors controlling quantitative resistance have contributed a great deal to the success in breeding resistant cultivars and their deployment [8]. Recent research has provided considerable evidence that the deployment of bacterial antagonists to *Xoo* might be an effective strategy, bringing about disease suppression by biological control [9].

To understand the epidemiology and ecology of *Xoo* pathogens and their potential for virulence change, various phenotypic characters as well as molecular markers have been used in studies of *Xoo* pathogen population structure [3, 4, 10, 11]. Rapid identification and classification of bacteria are normally carried out by morphology, nutritional requirements, antibiotic resistance, isozyme comparisons, phage sensitivity [7, 10, 12], and more recently DNA based methods, particularly rRNA sequences [13, 14], strain-specific fluorescent oligonucleotides [15], and the polymerase chain reaction (PCR) [12, 16]. Several repetitive elements found in the *Xoo* pathogen have been used as probes in restriction fragment length polymorphism (RFLP) analysis [17]. However, for the large number of samples needed for ecological and virulence studies, a simpler and cheaper technology is required. PCR is increasingly becoming an important tool in population biology, because of its simplicity and potential to rapidly screen a large number of samples with a minimal amount of DNA. 

In West Africa several *Xoo* genetic studies have been conducted and different *Xoo* pathotypes identified but little information is available on *Xoo* virulence genotypes population structure and distribution [10, 11, 18]. The virulence pathotypes of several *Xoo *isolates from West African countries based on cultivars reactions have been determined [4, 5, 19]. The main goal of this study is to determine *Xoo* virulence genotypes using the characterized *Xoo* isolates virulence pathotypes identified by Onasanya et al. [4] using random amplified polymorphic DNA polymerase chain reaction (RAPD-PCR) assays. The identification and differentiation of different *Xoo* virulence genotypes and distribution in West Africa would greatly help rice breeding improvement programs aiming at the effective development of rice cultivars with durable resistance to BLB disease.

## 2. Materials and Methods

### 2.1. Research Location

Bacterial isolate propagation and molecular PCR analysis were carried out at Central Biotechnology Laboratory, International Institute of Tropical Agriculture (IITA), Ibadan, Nigeria. This study was conducted between February and May 2009. 

### 2.2. Bacterial Isolates

Fifty *Xanthomonas oryzae *pv.* oryzae *(*Xoo*) isolates (Table 1) used in this study were from Onasanya et al. [4]. The identity of all the fifty *Xoo* isolates had been confirmed by oxidative biochemical test as well as their virulence pathotypes [4]. 

### 2.3. Isolates Propagation

BLB isolates were first propagated using a modified procedure developed by Onasanya et al. [18]. Nutrient broth (75 mL; pH 7.5) was prepared inside a 100 mL conical flask. Each *Xoo* isolate (100 *μ*L) from storage was transferred into 50 mL of nutrient broth and kept under constant shaking at 30°C for 24 hours for bacterial growth. The bacterial cell was removed by centrifugation, washed with 0.1 mM Tris-EDTA (pH 8.0), and kept at −20°C for DNA extraction.

### 2.4. Genomic DNA Extraction

DNA extraction was according to Onasanya et al. [20] and Onasanya et al. [18] with some modification. 0.3 g of washed bacterial cell was suspended in 200 *μ*L of cetyltrimethylammonium bromide (CTAB) buffer (50 mM Tris, pH 8.0; 0.7 mM NaCl; 10 mM EDTA; 2% hexadecyltrimethylammonium bromide; 0.1% 2-mercaptoethanol), followed by 100 *μ*L of 20% sodium dodecyl sulfate, and incubated at 65°C for 20 min. DNA was purified by two extractions with chloroform and precipitated with −20°C absolute ethanol. After being washed with 70% ethanol, the DNA was dried and resuspended in 200 *μ*L of sterile distilled water. DNA concentration was measured using DU-65UV spectrophotometer (Beckman Instruments Inc., Fullerto, CA, USA) at 260 nm. DNA quality was checked on a 1% agarose gel in Tris-acetate-EDTA (TAE) buffer (45 mM Tris-acetate, 1 mM EDTA, pH 8.0) after electrophoreses.

### 2.5. RAPD-PCR Analysis

This analysis was performed according to Onasanya et al. [20]. DNA primers used were purchased from Operon Technologies (Alameda, CA, USA) and each was ten nucleotides long. Two concentrations of each DNA (25 and 95 ng per reaction) were used to test reproducibility and eliminate sporadic amplification products from the analysis. Sixty primers (OPP, OPQ, OPR, OPS, OPT, OPV, OPX, and OPY series) were screened with DNA of two *Xoo* isolates (Virulence,* Vr,* and mildly virulence, *MVr, *isolates) for their ability to amplify the *Xoo* genomic DNA. Primers that gave useful polymorphisms were selected and used in amplifying the DNA from all *Xoo *isolates. Amplification was performed in 25 *μ*L reaction mixture consisting of genomic DNA; reaction buffer (Promega); 100 *μ*M each of dATP, dCTP, dGTP, and dTTP; 0.2 *μ*M Operon random primer; 2.5 *μ*M MgCl_2_, and 1U of Taq polymerase (Boehringer, Germany). A single primer was used in each reaction. Amplification was performed in a Thermowell microtiter plate (Costa Corporation) using an MJ Research Programmable Thermal Controller. The cycling program was (i) 1 cycle of 94°C for 3 min; (ii) 45 cycles of 94°C for 1 min for denaturation, 40°C for 1 min for annealing of primer, and 72°C for 2 min for extension; and (iii) a final extension at 72°C for 7 min. Amplification products were maintained at 4°C until electrophoresis.

### 2.6. Electrophoresis of PCR Products

The amplification products were resolved by electrophoresis in a 1.4% agarose gel using Tris-acetate-EDTA (TAE) buffer (45 mM Tris-acetate, 1 mM EDTA, pH 8.0) at 100 V for 2 h. A 1 kb ladder (Life Technologies, Gaithersburg, MD, USA) was included as molecular size marker. Gels were visualized by staining with ethidium bromide solution (0.5 *μ*g/mL) and banding patterns were photographed over UV light using UVP-computerized gel photo documentation system.

### 2.7. Cluster Analysis

Positions of scorable amplified DNA bands were transformed into a binary character matrix (“1” for the presence and “0” for the absence of a band at a particular position). Pairwise distance matrices were compiled by the Numerical Taxonomy System (NTSYS) 2.0 software [21] using the Jaccard coefficient of similarity [22]. Cluster dendrogram was created by unweighted pair-group method arithmetic (UPGMA) cluster analysis [23]. Principal component analysis with GGE biplot was carried out on 50 *Xoo* isolates using genetic data generated from twelve Operon primers [24].

## 3. Results and Discussion

Genetic analysis of fifty *Xanthomonas oryzae *pv* oryzae* (*Xoo*) isolates from West Africa has been carried out. After screening of 60 Operon primers with genomic DNA of two *Xoo* isolates (virulent pathotype, *Vr*, and mildly virulent pathotype, *MVr*), only 12 primers gave reproducible polymorphism and useful genetic information that differentiated the fifty *Xoo* isolates. Amplification with the 12 primers generated 210 bands from which 136 (64.8%) was polymorphic (Table 2) with sizes ranging between 0.5 and 4.0 kb (Figure 1). Using the 136 RAPD markers (Table 2) in cluster and principal component analyses revealed two major (*Mta* and *Mtb*) molecular typing virulence genotypes among fifty *Xoo* isolates (Figures 2 and 3). *Mta* genotype was made up of 42 virulence (*Vr*) *Xoo* isolates with two subgroup genotypes (*Mta1* and *Mta2*). *Mta1* (*Vr1*) subgroup genotype was typical of 25 *Xoo* isolates with 50% occurrence in six countries (Niger, Benin Republic, Nigeria, Burkina Faso, Mali, and Guinea) (Table 3). *Mta2* (*Vr2*) subgroup genotype was typical of 17 *Xoo* isolates with 34% occurrence in three countries (Mali, Guinea, and The Gambia) (Table 3). *Mtb* genotype characterized 8 mildly virulence (*MVr*) *Xoo* isolates with 16% occurrence in five countries (Niger, Benin Republic, Nigeria, Burkina Faso, and Guinea) (Table 3). Thus in Niger, Benin Republic, Nigeria, and Burkina Faso molecular typing revealed the presence of *Mta1* (*Vr1*) and *Mtb* (*MVr*) *Xoo* genotypes; *Mta1 *(*Vr1*), and *Mta2 *(*Vr2*) genotypes in Mali; *Mta1 *(*Vr1*), *Mta2 *(*Vr2*), and *Mtb *(*MVr*) genotypes in Guinea; and *Mta2* (*Vr2*) genotype in The Gambia (Figure 4, Table 3).

Molecular basis for African *Xoo* virulence identification is a prerequisite to understanding the genetics of *Xoo* virulence population structure in West Africa and deployment of durable resistance cultivars [1, 2, 25]. The present study examined if the two *Xoo* virulence pathotypes (*Pta* and *Ptb*) obtained using phenotypic pathotyping by Onasanya et al. [4] could be confirmed using molecular approach. Molecular typing using random amplified polymorphic (RAPD) markers has revealed two major (*Mta* and *Mtb*) virulence genotypes among the 50 *Xoo* isolates in which *Mta* was virulence (*Vr*) and *Mtb* mildly virulence (*MVr*). This paper supports recent isozyme fingerprints of 30 *Xoo* isolates from 5 countries (Mali, Burkina Faso, Niger, Benin Republic, and Nigeria) in West Africa and molecular analysis of 25 *Xoo* isolates from East Africa that revealed two major genetic groups [10, 11, 26]. These two genotypes of *Xoo* virulence identified by molecular typing were very identical to* Xoo* virulence pathotypes (*Pta* and *Ptb*) obtained using phenotypic pathotyping indicating possible linkage and correlation between phenotypic pathotyping and molecular typing of *Xoo* virulence [25, 27]. Besides, in other studies more variation has been observed within *Xoo* populations rather than between populations which might possibly explain the *Mta1* and *Mta2* subgroups obtained in the present study [28]. Moreover, incongruent relationship between different methods has been previously observed whereas the present study observed similar dendrogram relationships with different methods [28].

The high distinction pattern of each isolates in this study suggests possible high level of genetic variation and frequent occurrence of mutants in *Xoo* isolates in different host cells [10, 29, 30]. The genetic analyses revealed that *Mta* virulence genotype might cover about 84% of BLB population across Niger, Benin Republic, Nigeria, Burkina Faso, Mali, the Gambia, and Guinea and possibly be responsible for most sporadic cultivars infestation and epidemics in these countries. Also, the existence of *Mta1* and *Mta2* subgroups was likely due to mutations and interactions among isolates and strains that originally constituted *Mta* genotype [11, 18, 29, 31]. Mtb genotype existed in over 16% of BLB population across Niger, Benin Republic, Nigeria, Burkina Faso, and Guinea and might be responsible for most sporadic cultivars infestation and epidemics in these countries. *Mta1* (*Vr1*) and *Mtb* (*MVr*) genotypes were found to exist in Niger, Benin Republic, Nigeria, and Burkina Faso; *Mta1 *and *Mta2* in Mali; *Mta1*, *Mta2*,and *Mtb* in Guinea; and *Mta2 *in The Gambia, suggesting possible* Xoo* pathogen migration between these countries and long-term *Xoo* pathogen survival [1, 4, 18]. 

Distinct phenotypes usually consist of isolates that are genetically less related and such identification of isolates using cultural and morphological techniques often lacks consistency and precision [4]. Molecular typing of *Xoo* virulence has proven particularly useful in situations where it is necessary to differentiate virulence among two or more bacterial pathogens [18, 20, 27]. In the current study, it was discovered that identification of virulence in *Xoo* depends on different host origins and occurrence of mutants. For instance, *Mta* virulence genotype might cover about 84% of BLB population across Niger, Benin Republic, Nigeria, Burkina Faso, Mali, The Gambia, and Guinea, and *Mtb* genotype existed in over 16% of BLB population across Niger, Benin Republic, Nigeria, Burkina Faso, and Guinea, but isolates virulence distributions vary within subgroups. Based on phylogenetic study, it was discovered that after prolonged season-to-season interactions among isolates of *Mta* or *Mtb* genotype in different cultivated rice and weed hosts, different subgroup virulence genotypes (*Mta1* and *Mta2*) may emerge as a result of mutation [18, 20, 30]. The emerged subgroup virulence genotypes might result in occurrence of highly virulent isolates and strains with very broad interaction and pathogenicity across wide range of cultivated rice varieties across West African countries. 

## 4. Conclusions

The present molecular study of *Xoo* virulence identified two major *Xoo* virulence genotypes (*Mta* and *Mtb*) and two subgroups (*Mta1* and *Mta2*). Existence of different Xoo virulence genotypes suggests high level of *Xoo* pathogen interaction with host cells and mutation. The study revealed possible linkage between *Xoo* virulence pathotype and *Xoo* virulence genotype. Difference *Xoo* virulence genotypes were known to exist within country and there was evidence of *Xoo* pathogen migration between countries. Durable resistance rice cultivars would need to overcome both *Mta* and *Mtb Xoo* virulence genotypes in order to survive after their deployment into different rice ecologies in West Africa.

## Figures and Tables

**Figure 1:** DNA fingerprinting patterns of 50 *Xanthomonas oryzae *pv.* oryzae *(*Xoo*) isolates using OPS-08 random amplified polymorphic DNA primer. M: 1kb molecular size marker; kb: kilobase pair. *Xoo* isolates: 1 = XN-1; 2 = XN-2; 3 = XN-3; 4 = XN-4; 5 = XN-5; 6 = XN-6; 7 = XB-7; 8 = XB-8; 9 = XB-9; 10 = XB-10; 11 = XB-11; 12 = XNG-12; 13 = XNG-13; 14 = XNG-14; 15 = XNG-15; 16 = XNG-16; 17 = XBF-17; 18 = XBF-18; 19 = XBF-19; 20 = XBF-20; 21 =X BF-21; 22 = XBF-22; 23 = XM-23; 24 = XM-24; 25 = XM-25; 26 = XM-26; 27 = XM-27; 28 = XM-28; 29 = XM-29; 30 = XM-30; 31 = XG-31; 32 = XG-32; 33 = XG-33; 34 = XG-34; 35 = XG-35; 36 = XG-36; 37 = XG-37; 38 = XG-38; 39 = XG-39; 40 = XG-40; 41 = XTG-41; 42 = XTG-42; 43 = XTG-43; 44 = XTG-44; 45 = XTG-45; 46 = XTG-46; 47 = XTG-47; 48 = XTG-48; 49 = XTG-49; 50 = XTG-50.

**Figure 2:** Molecular typing of 50 *Xanthomonas oryzae *pv.* oryzae* (*Xoo*) virulence as revealed by 136 random amplified polymorphic DNA markers. *Mta*: molecular type a; *Mtb*: molecular type b; *Vr*: virulence; *MVr*: mildly virulence. *Xoo* isolates: 1 = XN-1; 2 = XN-2; 3 = XN-3; 4 = XN-4; 5 = XN-5; 6 = XN-6; 7 = XB-7; 8 = XB-8; 9 = XB-9; 10 = XB-10; 11 = XB-11; 12 = XNG-12; 13 = XNG-13; 14 = XNG-14; 15 = XNG-15; 16 = XNG-16; 17 = XBF-17; 18 = XBF-18; 19 = XBF-19; 20 = XBF-20; 21 = XBF-21; 22 = XBF-22; 23 = XM-23; 24 = XM-24; 25 = XM-25; 26 = XM-26; 27 = XM-27; 28 = XM-28; 29 = XM-29; 30 = XM-30; 31 = XG-31; 32 = XG-32; 33 = XG-33; 34 = XG-34; 35 = XG-35; 36 = XG-36; 37 = XG-37; 38 = XG-38; 39 = XG-39; 40 = XG-40; 41 = XTG-41; 42 = XTG-42; 43 = XTG-43; 44 = XTG-44; 45 = XTG-45; 46 = XTG-46; 47 = XTG-47; 48 = XTG-48; 49 = XTG-49; 50 = XTG-50.

**Figure 3:** Principal component analysis that revealed subgroup virulence genotypes among 50 *Xanthomonas oryzae *pv.* oryzae* isolates using genetic data generated from twelve random amplified polymorphic DNA (RAPD) primers.

**Figure 4:** *Xanthomonas oryzae* pv. *oryzae* isolates virulence genotype population structure status in West Africa. *Mta*: molecular type a; *Mtb*: molecular type b; *Vr*: virulence; *MVr*: mildly virulence. Country: C1: Niger; C2: Benin Republic; C3: Nigeria; C4: Burkina Faso; C5: Mali; C6: Guinea; C7: The Gambia.

**Table 1:** Identity of *Xanthomonas oryzae *pv.* oryzae* isolates used for the study.

S/N	Isolates codes∗	Host plant	Country
1	XN-1	D52-37	Niger
2	XN-2	D52-37	Niger
3	XN-3	IR15296829	Niger
4	XN-4	IR15296829	Niger
5	XN-5	WITA 8	Niger
6	XN-6	WITA 8	Niger
7	XB-7	Local	Benin
8	XB-8	Local	Benin
9	XB-9	Local	Benin
10	XB-10	Local	Benin
11	XB-11	Local	Benin
12	XNG-12	WITA9	Nigeria
13	XNG-13	WITA9	Nigeria
14	XNG-14	WITA 4	Nigeria
15	XNG-15	WITA 4	Nigeria
16	XNG-16	WITA 8	Nigeria
17	XBF-17	TS2	Burkina Faso
18	XBF-18	TS2	Burkina Faso
19	XBF-19	FKR14	Burkina Faso
20	XBF-20	FKR19	Burkina Faso
21	XBF-21	FKR14	Burkina Faso
22	XBF-22	Chinese	Burkina Faso
23	XM-23	Adventices	Mali
24	XM-24	Kogoni	Mali
25	XM-25	Kogoni	Mali
26	XM-26	Kogoni	Mali
27	XM-27	Kogoni	Mali
28	XM-28	Kogoni	Mali
29	XM-29	Jamajigi	Mali
30	XM-30	Nionoka	Mali
31	XG-31	Weed	Guinea
32	XG-32	Weed	Guinea
33	XG-33	Weed	Guinea
34	XG-34	Local	Guinea
35	XG-35	Local	Guinea
36	XG-36	Local	Guinea
37	XG-37	Local	Guinea
38	XG-38	Local	Guinea
39	XG-39	Local	Guinea
40	XG-40	Local	Guinea
41	XTG-41	Local	The Gambia
42	XTG-42	Local	The Gambia
43	XTG-43	Local	The Gambia
44	XTG-44	Local	The Gambia
45	XTG-45	Local	The Gambia
46	XTG-46	Local	The Gambia
47	XTG-47	Local	The Gambia
48	XTG-48	Local	The Gambia
49	XTG-49	Weed	The Gambia
50	XTG-50	Weed	The Gambia

^*^ *Xanthomonas oryzae *pv.* oryzae* isolates obtained from [4].

**Table 2:** Oligonucleotide primers that showed genetic discrimination among the *Xanthomonas oryzae *pv.* oryzae* isolates using random amplified polymorphic DNA polymerase chain reaction analysis.

Operon primer	Nucleotide sequence 5′ to 3′	No. of fragments amplified	No. of polymorphic bands	% polymorphism
OPP-17	TGACCCGCCT	18	16	88.9
OPP-18	GGCTTGGCCT	14	11	78.6
OPR-07	ACTGGCCTGA	20	11	55.0
OPS-08	TTCAGGGTGG	23	13	56.5
OPS-10	ACCGTTCCAG	20	13	65.0
OPS-13	GTCGTTCCTG	16	9	56.3
OPT-09	CACCCCTGAG	16	10	62.5
OPT-12	GGGTGTGTAG	13	7	53.8
OPT-15	GGATGCCACT	18	10	55.6
OPV-05	TCCGAGAGGG	19	12	63.2
OPY-06	AAGGCTCACC	16	11	68.8
OPY-08	AGGCAGAGCA	17	13	76.5

Total		210	136	64.8

**Table 3:** *Xanthomonas oryzae *pv.* oryzae* isolate group, virulence, and distribution relative to country of origin.

Typing	Main group	Subgroup	Virulence	Isolate origin and distribution							% Occurrence
				Niger	Benin	Nigeria	Burkina Faso	Mali	Guinea	The Gambia	
Pathotype∗	*Pta*	*Pta*1	*Vr*	—	—	—	4	1	4	1	20
		*Pta*2	*Vr*	3	—	—	—	—	1	4	16
		*Pta*3	*Vr*	—	2	3	1	2	3	—	22
	*Ptb*	*Ptb*1	*MVr*	2	2	1	1	1	1	2	20
		*Ptb*2	*MVr*	1	1	1	—	4	1	3	22

Molecular type	*Mta*	*Mta*1	*Vr*1	4	3	3	5	7	3	—	50
		*Mta*2	*Vr*2	—	—	—	—	1	6	10	34
	*Mtb*	—	*MVr*	2	2	2	1	—	1	—	16

^*^[4]*; Pta*: pathotype a; *Ptb*: pathotype b; *Mta*: molecular type a; *Mtb*: molecular type b; *Vr*: virulence; *MVr*: mildly virulence.
